The article "Corporate governance, technological innovation, and corporate performance: Evidence from China" was retracted in 2025. Reasons: unreliable results or conclusions; concerns about the authorship.

# Corporate governance, technological innovation, and corporate performance: Evidence from China

**DOI:** 10.1016/j.heliyon.2024.e31459

**Published:** 2024-05-16

**Authors:** Yinlong Ma, Nur Syafiqah Binti A. Rahim, Siti Aisyah Bt Panatik, Ruirui Li

**Affiliations:** a School of Human Resources Development & Psychology, Universiti Teknologi Malaysia, Johor Bahru, Johor, 81300, Malaysia; b Xinhua College, Ningxia University, Yinchuan, Ningxia, 750021, China

**Keywords:** Corporate governance, Technological innovation, Corporate performance

## Abstract

Corporate governance plays an important role in achieving high-quality economic development and sustainable corporate development. In recent years, as listed companies face increasing challenges in social responsibility issues such as environmental pollution and financial fraud, corporate governance has received widespread attention from academics and practitioners. In particular, technological innovation has attracted much attention to the development of enterprises. This paper also explores the intermediary mechanism of technological innovation based on the output measurement method of technological innovation. This study selected data from companies listed on the A-share main board of the Shanghai and Shenzhen Stock Exchanges in China from 2012 to 2022, aiming to explore the relationship between corporate governance and corporate performance. At the same time, we further analyzed the impact of corporate governance on corporate performance based on the mediating role of technological innovation. The research results show that equity balance degree, board size, and executive incentives all have a positive impact on corporate performance. Technological innovation has a certain mediating effect on independent variables (equity balance degree, board size, and executive incentives) and corporate performance. This study clarifies the controversy about the relationship between corporate governance and corporate performance and deepens the understanding of this relationship. It also provides empirical support for listed companies to pay attention to and improve corporate governance levels and enhance innovation capabilities. By exploring the interplay between governance mechanisms, innovation processes, and performance outcomes, researchers can gain a deeper understanding of how organizations can leverage governance practices to drive innovation-led growth and sustainable success.

## 1 Introduction

Corporate performance is significant to investors, shareholders, and stakeholders. Especially for investors, corporate performance is an important basis for them to choose investment companies[1]. Evidence shows that corporate governance and technological innovation are important factors affecting corporate performance[2,3]. Enterprise ESG construction has a significant positive impact on regional green economy efficiency [64]. Moreover, digital transformation influences business decisions through green technology innovation [4].

The article "Corporate governance, technological innovation, and corporate performance: Evidence from China" was retracted in 2025. Reasons: unreliable results or conclusions; concerns about the authorship.

Previous literature discusses the impact of corporate governance on technological innovation, corporate performance, corporate sustainable development, tax policy, and corporate value from the perspectives of ownership structure, board governance, management governance, institutional investors, and venture capital[5]. Corporate governance is one of the critical elements of corporate performance that can help to improve the long-term value of corporate, which will enhance corporate performance[6,7]

China's economy has entered a new era in which growth is slowing down, quality is light, volume is heavy and strength is heavy, which also puts forward higher requirements for corporate governance [7]. The Chinese corporate governance system is mainly characterized by the dominance of one share, therefore, the agency problem is serious[8]. It is very important to improve the efficiency of corporate governance in China to reduce agency costs.

Previous studies have examined the relationship between corporate governance and corporate performance, and the relationship between corporate governance and technological innovation based on agency theory. The literature on internal controls and corporate technological innovation, particularly focusing on Chinese listed companies, addresses the intricate relationship between internal control mechanisms and the fostering of innovation within corporate entities[9]. The literature on the relationship between corporate governance and the cost of equity during the ISIS era in Iraq underscores the critical role of governance mechanisms in shaping investor perception, market dynamics, and the cost of capital in a challenging and volatile environment[10]. However, previous studies have drawn inconsistent conclusions on the relationship between corporate governance and corporate performance, corporate governance, and technological innovation [11].

From the particularity of the country's system and the characteristics of the environment view, the current literature research on the relationship between corporate governance and corporate performance lacks consideration [12]. The organic embedding of party organizations in the corporate governance system through two-way entry and cross-appointment is where the institutional strength of Chinese enterprises lies and is a crucial element of corporate governance modernization[13]. China's corporate governance structure has its particularity. Since 2015, China's ownership structure has changed from centralized to decentralized[14]. Considering the importance of China's A-share listed companies to China's GDP, this study takes China's A-share listed companies as the research background to explore the relationship between corporate governance, technological innovation, and corporate performance, which will be used to fill the current research gap in the study.

The article "Corporate governance, technological innovation, and corporate performance: Evidence from China" was retracted in 2025. Reasons: unreliable results or conclusions; concerns about the authorship.

There is no research on the role of technological innovation in corporate governance and corporate performance[15]. This study attempts to explain the role of technological innovation in the relationship between corporate governance and corporate performance from a classical (agency theory) perspective. Understanding the relationship between corporate governance, technological innovation, and corporate performance aids in the discovery of evidence that technological innovation acts as a mediator variable [16].

This study focuses on resolving the gaps in previous research by exploring the interrelationship between corporate governance, technological innovation, and corporate governance. This research endeavours to provide empirical evidence regarding how the implementation and effectiveness of internal controls influence the innovation activities of Chinese firms, particularly in the context of rapidly evolving technological landscapes and the competitive pressures of the global market. This study considers the key variables affecting corporate governance and examines the mediating effect of technological innovation between corporate governance and corporate performance for Chinese A-share listed companies. The reason why this study selects China as the research context lies in that China is playing an increasingly important role in the world economy, in which A-share listed Chinese companies are receiving more attention from both Chinese investors and foreign investors, who cares a lot about the corporate governance issue relating closely to technological innovation and corporate performance.

This study mainly draws on a famous corporate governance scholar, Li Weian's definition of corporate governance. Narrowly defined corporate governance refers to a supervisory and balancing mechanism of owners (mainly shareholders) over operators. Its main feature is the internal governance of the corporate governance structure composed of shareholder meetings, board of directors, supervisory board, and management. This study mainly explores the impact of internal governance mechanisms on corporate performance, therefore equity balance, board size, and executive equity incentives in internal mechanisms are selected to measure the level of internal corporate governance of listed companies.

The article "Corporate governance, technological innovation, and corporate performance: Evidence from China" was retracted in 2025. Reasons: unreliable results or conclusions; concerns about the authorship.

The definition of technological innovation is quite complex, the following indicators are generally used to measure technological innovation in academic research.

(1) R&D investment: R&D expenditure is one of the most direct indicators for measuring technological innovation. The greater the investment of enterprises or countries in research and development activities, the higher their emphasis on technological innovation.
(2) Number and quality of patents: The number and quality of patents are important indicators for measuring technological innovation. The number of patents owned by a company, as well as the technological content and innovation level of these patents, can reflect its technological innovation strength.
(3) New product development: The development and launch of new products can be seen as a technological innovation activity. The quantity, quality, and market influence of new products can be used as indicators to measure technological innovation.

This study mainly uses the ratio of R&D investment to revenue to measure technological innovation.

This study is the first research on the correlation among corporate governance, technical innovation and corporate performance of A-share listed company, which will make a detailed examination of the specific functions and impacts of corporate government and technical innovation on corporate performance and make an original contribution to the complete understanding of the correlation of these 3 variables.

## 2 Literature review

This part mainly introduces the theoretical basis related to the research, and combing the literature according to the research theme, laying a foundation for the writing of the paper.

### 2.1 Theoretical background

The basic theory of this study reviews and discusses the theories related to agency. The principal-agent theory is one of the most significant advancements in contract theory to occur within the past three decades[17]. It was developed in the late 1960s and early 1970s by a group of economists who had conducted in-depth research on the information asymmetry and incentive issues that plagued corporates [18]. The study of how the principal comes up with the best possible contract to motivate the agent in a setting where there are competing interests and unequal amounts of information is the primary objective of principal-agent theory[19].

### 2.2 Literature review and hypothesis

#### 2.2.1 Equity balance degree and corporate performance

With China's reform of non-tradable shares, the equity factor has gradually impacted corporate performance [20]. The better the corporate performance, the bigger the degree of equity balance, the more fairly dispersed equity, and the lower the percentage of ownership held by the largest shareholder[21]. When a corporation's largest shareholder has a small shareholding percentage, the amount of stock balance has little bearing on how well the corporation performs. If a certain threshold value is exceeded, the degree of equity balance has a positive effect on company performance[22]. According to Chen [23] research on the top five shareholders' equity checks and balances, these checks and balances have a moderating effect on company performance. Some people think that the presence of fair checks and balances contributes to improving the effectiveness of internal control and has a significant positive effect on corporate performance[24].

The article "Corporate governance, technological innovation, and corporate performance: Evidence from China" was retracted in 2025. Reasons: unreliable results or conclusions; concerns about the authorship.

Thus, based on the discussion, the researcher believes the relationship is positive between equity balance degree and corporate performance leading to hypothesis 1:

Hypothesis 1 There is a significant relationship between equity balance degree and the corporate performance of China-listed companies on A-share.

#### 2.2.2 Board size and corporate performance

Tran et al. [25]identified board size, gender diversity on the board, group ownership, and the existence of sustainability committees as important factors in determining a corporation's sustainable development. Performance in terms of sustainability is positively connected with the size of the board and the frequency of board meetings. And in the long run, the board's capital structure promotes low-carbon sustainable development [66], [67]. According to Al-Qatanani and Siam [26] research, there is a positive association between board features and corporate performance, suggesting that a more successful board is linked to better management behaviour monitoring. Higher board size, ROA, and Tobin's Q have a positive and significant impact on corporate performance, which aids in strengthening the decision-making process, according to Neralla [27] 's research. Effective board management and high corporate performance have a strong positive association[28].

As a result of the conversation, the researcher believes the relationship positive between board size and corporate performance leading to hypothesis 2:

Hypothesis 2 There is a significant relationship between board size and corporate performance of China-listed companies on A-share.

#### 2.2.3 Executive equity incentive and corporate performance

Jensen and Meckling [29] believed from the perspective of interest convergence that equity incentives could further promote corporate performance by making managers' interests the same as shareholders' interests. According to the agency theory, equity incentives can help managers get residual income, to reduce the contradiction between managers and owners[30]. Equity incentives can force managers to make more accurate decisions from the perspective of their interests, it will reduce overinvestment and underinvestment, and other problems. In addition, there is also a relationship between equity incentive intensity and corporate performance. In corporations implementing equity incentives, with the increase of equity incentive intensity, corporate performance will further increase[31].

The article "Corporate governance, technological innovation, and corporate performance: Evidence from China" was retracted in 2025. Reasons: unreliable results or conclusions; concerns about the authorship.

Thus, based on the discussion, the researcher believes the relationship positive between executive equity incentives and corporate performance leading to hypothesis 3:

Hypothesis 3 There is a significant relationship between executive equity incentives and the corporate performance of China-listed companies on A-share.

#### 2.2.4 Equity balance degree and technological innovation

The direct connection between corporate governance and technological innovation for companies listed on the A-share main board in China revolves around board composition, executive incentives, regulatory dynamics, access to capital, and intellectual property protection. Addressing these specific challenges within the context of China's unique market environment is essential for driving innovation-led growth and sustainable development.

The equity balance degree refers to the distribution and restriction relationship of power within the company. The equity balance degree is crucial to the development of an enterprise. It can effectively avoid excessive concentration of power within the company, thereby ensuring the company's stability and sustainable development. Technological innovation is an important driving force for enterprise development. It can improve the competitiveness and market share of enterprises. Based on the perspective of agency theory, based on moderate concentration of ownership, the equity balance degree has a significant positive correlation with technological innovation and corporate performance [32]. Another view is that the equity balance degree is negatively correlated with technological innovation. This is based on the perspective of innovation theory, which believes that the equity balance degree will increase the internal conflicts and coordination costs of enterprises, reduce the innovation efficiency and quality of enterprises, and affect the innovation power and capabilities of enterprises [33]. In addition, the relationship between equity balance degree and technological innovation is complex and is affected and regulated by a variety of factors, such as industry competitiveness, ownership nature, technological innovation risks, etc. Guo and Chen [34] introduced technological innovation as a mediating variable to analyze the relationship between ownership structure, technological innovation, and corporate performance and found that technological innovation partially mediates the impact of ownership structure on corporate performance.

The article "Corporate governance, technological innovation, and corporate performance: Evidence from China" was retracted in 2025. Reasons: unreliable results or conclusions; concerns about the authorship.

Thus, based on the discussion, the researcher believes the relationship is positive between equity balance degree and technological innovation leading to hypothesis 4:

Hypothesis 4 There is a significant relationship between equity balance degree and the technological innovation of China-listed companies on A-share.

#### 2.2.5 Board size and technological innovation

The board of directors serves as the primary organizational structure of modern corporations. Some scholars believe that the more members on the board of directors, the more complementary advantages can be formed, which can alleviate agency problems in the process of technological innovation[35]. However, some people believe that as the size of the board of directors increases, the efficiency of decision-making will be reduced, because there may be a “free rider” problem, which will inhibit investment in innovation corporate[36]. Zhao et al. [37] through regression analysis, it was determined that board size positively influences green innovation. The board of directors and the independent directors will have a significant favourable impact on corporate technological innovation[38]. The frequency of board meetings and the overall compensation of directors are both connected to how effectively technical innovation works, but the opposite is true for the number of shares that directors possess [39].

In light of the discussion, the researcher believes the relationship is positive between board size and technological innovation leading to hypothesis 5:

Hypothesis 5 There is a significant relationship between board size and technological innovation of China-listed companies on A-share.

#### 2.2.6 Executive equity incentive and technological innovation

Equity incentives and technological innovation have been the main topics of scholars' attention and research. The equity incentive can effectively link managers' interests, and the incentive impact will be better. According to several studies, the equity incentive raises the company's long-term worth[40]. Equity incentive is mainly to give managers certain equity to encourage managers to pay attention to the corporation's technological innovation activities from a long-term perspective [41]. Ma and Wan [42] investigated the impact of equity incentives on technological innovation and the findings indicated that equity incentives of listed companies can promote corporate technological innovation ability.

The article "Corporate governance, technological innovation, and corporate performance: Evidence from China" was retracted in 2025. Reasons: unreliable results or conclusions; concerns about the authorship.

Equity incentives can alleviate the principal-agent problem of corporations, promote managers to pursue long-term development, facilitate corporations to conduct external financing, and then provide financial support for technological innovation[43]. The option incentive of core technical staff has a big impact on innovation in industries that rely heavily on technology[44]. The new executive incentive system has a positive effect on the cost of equity through good governance. In particular, the incentive system of executive pay brings down the cost of equity by a lot[45]. As a result of the argument, the researcher feels that the executive equity incentive has a significance to technological innovation, leading to hypothesis 6:

Hypothesis 6 There is a significant relationship between executive equity incentives and the technological innovation of China-listed companies on A-share.

#### 2.2.7 The mediating role of technological innovation on the relationship between corporate governance and corporate performance

For the development of corporations' long-term interests, shareholders are more motivated to pay attention to the development of technological innovation of corporations, to bring long-term interests to shareholders themselves [66], [67]. Yuan and Song [46] show that there is an upside-down U-shaped relationship between ownership concentration and corporate performance and that corporate innovation is a key part of how corporate ownership dispersion improves corporate performance. Qin et al. [47] found that technological innovation has a mediating effect between ownership structure and corporate performance.

The board of directors is the main institution of internal governance of listed companies. It mainly supervises operators on behalf of shareholders in the daily operation and management of the corporation and makes decisions on the daily operation of the corporation [48]. The board of directors can build corporate R&D alliances through group alliances, hence the board of directors' participation in innovation outcomes is critical [49]. According to Xia et al. [50], larger boards of directors have greater knowledge levels, management skills, and decision-making abilities, which can help the company's technological innovation operations advance smoothly. To encourage corporate innovation, board size is crucial[51]. According to Di et al. [52] corporate management personnel have a significant influence on the choice to spend in R&D, which impacts corporate performance.

The article "Corporate governance, technological innovation, and corporate performance: Evidence from China" was retracted in 2025. Reasons: unreliable results or conclusions; concerns about the authorship.

There is an essential relationship between corporate technology innovation and corporate value[53]. Zuo [54] found that the share of major shareholders is positively related to technological innovation and corporate performance. Equilibrium is directly related to technological innovation and corporate performance. Part of the effect of ownership on corporate performance is mediated by innovative technology. According to Di et al. [52], technological innovation entirely mediates the diversification of board diversity and corporate performance. As a result, taking corporate technological innovation into account as an intermediate when examining the relationship between corporate governance and corporate performance will result in a more precise explanation[55].

Therefore, this study takes technological innovation as the intermediate variable to study. The following hypotheses 7–9 can be derived from the study presented above:

Hypothesis 7 Technological innovation in Chinese A-share listed companies has a mediating effect between equity balance degree and corporate performance.

Hypothesis 8 Technological innovation in Chinese A-share listed companies has a mediating effect between board size and corporate performance.

Hypothesis 9 Technological innovation in Chinese A-share listed companies has a mediating effect between executive equity incentive and corporate performance.

In short, based on the overall literature review, there is a seriously positive relationship between corporate governance, technological innovation and corporate performance.

## 3 Research design

In order to solve the research problem, the framework, structure and methods used to collect relevant data, analyze findings and draw conclusions are presented in this section.

### 3.1 Sample description and data sources

This study presents a comprehensive study on corporate governance, technological innovation, and corporate performance of Chinese A-share listed companies. The sample is mainly collected from 597 companies listed on the Chinese A-share, with a period of 5970 sample observations over 10 years from 2012 to 2021. The following kinds of company were not included in the study's sample selection method based on prior research literature:

(1) Eliminate the financial and real estate companies,
(2) Eliminate ST and * ST and sample period has been delisted corporate,
(3) To eliminate absence the key variables for five consecutive years corporate,
(4) The level of the corporate continuous variables were 1 % and 99 % points of shrinkage end processing.

The exclusion of financial and real estate companies is based on the following main reasons. (1) Differences in industry characteristics: the finance and real estate industries have unique characteristics compared to other industries. The profit model, risk management mechanism, and capital operation mode of the financial industry are very different from other industries. Similarly, the profit model and asset liability structure of the real estate industry also differ significantly from other industries. Therefore, studying financial and real estate companies may lead to increased sample heterogeneity, reducing the universality and reliability of research conclusions. (2) Data comparability: The financial and real estate industries may have significant differences in financial data and operating indicators compared to other industries, which can affect the comparability of research results. If financial and real estate companies are included in the research sample, it may introduce more noise, making the analysis of the relationship between corporate governance and corporate performance more complex. (3) Different research purposes: When studying the impact of corporate governance on corporate performance, it is usually hoped to obtain conclusions that are universally applicable to various industries. Due to their unique characteristics, the financial and real estate industries may require separate research and the use of specialized analytical frameworks and methods. Therefore, in order to maintain consistency and comparability of the research, it may be chosen to exclude companies from these special industries. (4) When selecting samples, this study drew on the standards currently used by scholars to select samples of A-share listed companies in China.

The article "Corporate governance, technological innovation, and corporate performance: Evidence from China" was retracted in 2025. Reasons: unreliable results or conclusions; concerns about the authorship.

Among them, corporate governance variables (equity balance degree, board size, executive equity incentive) and corporate performance variables are mainly collected from CSMAR (China Economic and Financial Research Database), and technological innovation data are mainly collected from the China patent database. However, some of the additional information for the study's control variables was gathered from the corporation's annual report and the China Securities Exchange Market.

### 3.2 Research model

Based on the research hypothesis, the following multiple linear regression model is constructed to examine the impact of corporate governance on corporate performance.

(1) $${\text{ROE}}_{i,t}=a_{0}+a_{1}Z_{i,t}+a_{2}{\text{BS}}_{i,t}+a_{3}{\text{EEI}}_{i,t}+a_{4}{\text{DTAR}}_{i,t}+a_{5}{\text{FS}}_{i,t}+a_{6}{\text{NPGR}}_{i,t}+\sigma_{i,t}+\varepsilon_{i,t}$$

(Equation (1) is set as abovementioned to examine the impact of corporate governance on corporate performance.)

Among them，ROE_i,t_ is corporate performance，Z_i,t_ is equity balance degree， BS_i,t_ is board size， EEI_i,t_ is executive equity incentive，DTAR_i,t_ is the asset-liability ratio、FS_i,t_ is the scale of the corporate, NPGR_i,t_ is the net profit growth rate，σ_i,t_ is the individual and time fixed effects, ε_i,t_ is the random disturbance term.

The article "Corporate governance, technological innovation, and corporate performance: Evidence from China" was retracted in 2025. Reasons: unreliable results or conclusions; concerns about the authorship.

### 3.3 Variable measures

Table 1 shows the study's sorting of explained variables, explanatory variables, mediating variables and control variables, and the methods to measure them according to the listed references in the table.

**Table 1:** Variable definition.

Variable		Variable Identifier	Variable Measurement
Explained Variable	Return on Equity	ROE	Annual net profit/closing net assets [65].
	Return on Total Assets	ROA	Net profit/total asset balance[56].
Explanatory Variables	Equity Balance Degree	Z	The total number of shares owned by the second through fifth-largest shareholders is divided by the number of shares owned by the largest shareholder. The more checks and balances there are to make sure things are fair, the higher the percentage[11].
	Board Size	BS	End of the year total number of directors[57].
	Executive Equity Incentive	EEI	Number of shares held by senior management [58].
Mediating Variable	Technological Innovation		R&D investment as a percentage of revenue [59,60].
Control Variables	Debt-To-Assets Ratio	DTAR	Total liabilities/total assets[22].
	Corporate Size	CS	Calculated using the natural logarithm of total assets[61].
	Net Profit Growth Rate	NOGR	Rate of increase in net profit[62].

## 4 Empirical analysis

According to the research model, this part mainly carries on the empirical analysis of the data, and discusses the relationship between the relevant variables.

### 4.1 Descriptive statistics

Table 2 shows the results of the empirical analysis of the data of variables in the 1st column.

**Table 2:** Descriptive statistics.

VarName	Obs	Mean	SD	Min	Median	Max
ROE	5970	0.0909	0.0682	−2.0580	0.0820	0.5010
ROA	5970	0.0573	0.0423	−0.3950	0.0490	0.3050
TI	5970	18.3392	1.3303	11.6904	18.2704	23.7483
Z	5970	0.7413	0.6091	0.0082	0.5448	3.9194
BS	5970	2.1244	0.1901	1.0986	2.1972	2.8904
EEI	5970	12.6814	6.5612	0.0000	14.9407	21.4847
DTAR	5970	0.3673	0.1793	0.0110	0.3550	0.9600
FS	5970	22.3077	1.1802	19.5440	22.1635	27.5470
NPGR	5970	0.4750	4.3741	−40.4240	0.1355	164.5670

**Table 3:** Correlation analysis.

	ROE	ROA	TI	Z	BS	EEI	DTAR	FS	NPGR
ROE	1								
ROA	0.811***	1							
TI	0.197***	0.070***	1						
Z	0.029**	0.085***	0.023*	1					
BS	0.052***	0.019*	0.133***	0.068***	1				
EEI	0.062***	0.136***	0.070***	0.239***	−0.052***	1			
DTAR	−0.002	−0.355***	0.335***	−0.119***	0.095***	−0.190***	1		
FS	0.154***	−0.040***	0.670***	−0.060***	0.185***	−0.107***	0.584***	1	
NPGR	0.125***	0.101***	0.001	−0.005	0.027**	−0.030**	0.032**	0.037***	1

Note: *, **, and *** represent significance at the 10 %, 5 %, and 1 % levels respectively.

The article "Corporate governance, technological innovation, and corporate performance: Evidence from China" was retracted in 2025. Reasons: unreliable results or conclusions; concerns about the authorship.

The average value of the corporate performance indicator ROE (return on equity) is 0.0909, and the standard deviation is 0.0682, indicating that the distribution of corporate return on equity in the sample is relatively concentrated, but there is also a certain degree of fluctuation. The mean value of ROA (return on total assets) is 0.0573 and the standard deviation is 0.0423. Compared with ROE, the volatility of ROA is slightly lower, but it also shows significant differences in return on assets between companies. The average value of technological innovation (TI) is 18.3392, and the standard deviation is 1.3303, indicating that the performance of sample enterprises in technological innovation is relatively consistent, but there are still certain differences. The average value of the equity balance degree (Z) is 0.7413, and the standard deviation is 0.6091, which shows that the equity structure varies greatly among the sample companies. The mean value of board size (BS) is 2.1244 and the standard deviation is 0.1901, indicating that the board size of the sample companies is relatively stable, but there is still a certain degree of variability. The mean value of executive equity incentives (EEI) is 12.6814 and the standard deviation is 6.5612, indicating that there are large differences in executive equity incentives among sample companies. The average value of the debt-to-asset ratio (DTAR) is 0.3673, and the standard deviation is 0.1793, showing the differences in financial leverage among sample companies. The mean value of firm size (FS) is 22.3077 and the standard deviation is 1.1802, indicating that the sample firms are relatively uniform in size, but there are still certain size differences. The mean value of the net profit growth rate (NPGR) is 0.4750, but the standard deviation is 4.3741. This large standard deviation points out the great differences in the profitability growth of sample companies.

In summary, the descriptive statistical results reveal the distribution characteristics and differences of sample companies in terms of ownership structure, board size, executive incentives, technological innovation, and financial indicators. These differences provide information for subsequent statistical analysis and hypothesis testing. foundation.

### 4.2 Correlation analysis

The correlation coefficient between ROE and ROA is 0.811, and it is significant at the 1 % significance level (***), indicating that the return on net assets of the company is highly positively related to the return on total assets, that is, the performance of these two The indicators generally move in the same direction, which is expected since they are both measures of a company's profitability.

The article "Corporate governance, technological innovation, and corporate performance: Evidence from China" was retracted in 2025. Reasons: unreliable results or conclusions; concerns about the authorship.

The correlation coefficients between technological innovation (TI) and ROE and ROA are 0.197 and 0.070 respectively, both significant at the 1 % significance level, indicating that technological innovation is positively related to corporate performance, although the degree of correlation is different. This may indicate that technological innovation plays a positive role in improving corporate performance.

The correlation coefficients between ownership structure (Z) and ROE and ROA are 0.029 and 0.085 respectively, which are significant at the 5 % and 1 % significance levels respectively. This indicates that there is a weak positive correlation between the degree of equity checks and balances and corporate performance. relation.

The correlation coefficient between board size (BS) and ROE is 0.052, which is significant at the 1 % significance level, and the correlation coefficient with ROA is 0.019, which is significant at the 10 % significance level.

The correlation coefficients between executive equity incentives (EEI) and ROE and ROA are 0.062 and 0.136 respectively, both significant at the 1 % significance level. This shows that executive equity incentives are positively related to corporate performance, possibly because of equity incentives, and stimulate the enthusiasm of management, thereby improving the profitability of the company as indicated in Table 3.

### 4.3 Regression

To test the collinearity of the model, this article uses the variance inflation factor to test. As can be seen from Table 4 above, the VIF of all variables is less than 5, indicating that the model does not have obvious multicollinearity problems.

**Table 4:** Multicollinearity test.

	VIF	1/VIF
DTAR	1.5656	0.6387
FS	1.5592	0.6413
EEI	1.0950	0.9132
Z	1.0756	0.9297
BS	1.0457	0.9563
NPGR	1.0025	0.9975
Mean VIF	1.2240	.

As indicated in Table 5 above, the impact coefficient of equity balance degree (Z) on ROE is 0.0071, which is significant at the 1 % significance level, indicating that for every unit increase in the degree of checks and balances in the ownership structure, the company's return on net assets increases by 0.71 on average. percentage point. The coefficient of board size (BS) is 0.0184, which is significant at the 5 % significance level, indicating that for every unit increase in board size, ROE increases by 1.84 percentage points on average. The coefficient of executive equity incentives (EEI) is 0.0005, which is significant at the 5 % significance level, implying that executive equity incentives are positively related to corporate performance.

The article "Corporate governance, technological innovation, and corporate performance: Evidence from China" was retracted in 2025. Reasons: unreliable results or conclusions; concerns about the authorship.

**Table 5:** Regression of independent variables on ROE.

	(1)
	ROE
Z	0.0071***
	(2.6830)
BS	0.0184**
	(2.4292)
EEI	0.0005**
	(2.4331)
DTAR	0.0176*
	(1.8511)
FS	0.0041*
	(1.6838)
NPGR	0.0023***
	(13.8970)
_cons	−0.0505
	(-0.9657)
N	5970
F	17.8270
Firm	Yes
Year	Yes
R^2^	0.0475

Note: *, **, and *** represent significance at the 10 %, 5 %, and 1 % levels respectively.

As shown in Table 6 above, the coefficient of equity balance degree (Z) on technological innovation (TI) is 0.1098, which is significant at the 1 % significance level, and the t value is 5.5585. This shows that the equity balance degree is positively related to technological innovation, and the relationship is significant. Specifically, for every unit increase in the equity balance degree, the level of technological innovation increases by an average of 0.1098 units (see Table 7).

**Table 6:** Regression of independent variables on TI.

	(1)
	TI
Z	0.1098***
	(5.5585)
BS	0.1378**
	(2.4473)
EEI	0.0053***
	(3.2468)
DTAR	−0.0540
	(-0.7647)
FS	0.7116***
	(39.3884)
NPGR	−0.0038***
	(-3.1684)
_cons	1.7666***
	(4.5536)
N	5970
F	709.0251
Firm	Yes
Year	Yes
R^2^	0.6650

Note: *, **, and *** represent significance at the 10 %, 5 %, and 1 % levels respectively.

**Table 7:** Robustness test.

	(1)	(2)
	ROA	ROA
TI		0.0102***
		(10.4490)
Z	0.0039***	0.0028**
	(2.7609)	(1.9895)
BS	0.0109***	0.0095**
	(2.6972)	(2.3736)
EEI	0.0004***	0.0004***
	(3.5560)	(3.1251)
DTAR	−0.0699***	−0.0694***
	(-13.7664)	(-13.7948)
FS	0.0047***	−0.0025*
	(3.6274)	(-1.7250)
NPGR	0.0012***	0.0013***
	(14.0354)	(14.6150)
_cons	−0.0470*	−0.0649**
	(-1.6833)	(-2.3457)
N	5970	5970
F	36.1420	41.3911
Firm	Yes	Yes
Year	Yes	Yes
R^2^	0.0919	0.1100

Note: *, **, and *** represent significance at the 10 %, 5 %, and 1 % levels respectively.

The coefficient of board size (BS) is 0.1378, which is significant at the 5 % significance level, and the t value is 2.4473, indicating that board size has a significant positive impact on technological innovation. This may be because larger boards may have more resources and diversity, thereby promoting technological innovation.

The coefficient of executive equity incentives (EEI) is 0.0053, which is significant at the 1 % significance level, and the t value is 3.2468, showing that executive equity incentives are positively related to technological innovation. This may mean that when executives own shares in a company, they are more likely to drive technological innovation in the company to increase the company's long-term value.

### 4.4 Robustness test

To ensure the correctness of the research results of corporate governance on corporate performance, this study mainly used the method of replacing the dependent variable to conduct a robustness test.

The article "Corporate governance, technological innovation, and corporate performance: Evidence from China" was retracted in 2025. Reasons: unreliable results or conclusions; concerns about the authorship.

To avoid the contingency of the regression results, this article will replace the explanatory variable with ROA and conduct the regression again. The results are shown in Table 6. In column (1), the impact coefficient of equity balance degree (Z) on ROA is 0.0039, which is significant at the 1 % significance level. It means that for every unit increase in the equity balance degree, the return on total assets increases by 0.39 on average. percentage points. The coefficient of board size (BS) is 0.0109, which is significant at the 1 % significance level, indicating that board size also has a positive impact on ROA. The coefficient of executive equity incentives (EEI) is 0.0004, which is significant at the 1 % significance level, showing that executive equity incentives are positively related to ROA.

In column (2), the coefficient of technological innovation (TI) on ROA is 0.0102, both of which are significant at the 1 % significance level. This shows that technological innovation has a significant positive impact on corporate performance, that is, an increase in the level of technological innovation can significantly increase a company's return on net assets and return on total assets.

The direct impact coefficient of equity balance degree (Z) on ROA is significant at the 5 % significance level. This may indicate that part of the impact of ownership structure is realized through the intermediary variable of technological innovation. That is, the equity balance degree may improve corporate performance by promoting technological innovation. Board size (BS) has a positive impact on and is significant at the 5 % significance level. This shows that the size of the board of directors may directly affect corporate performance, and may also indirectly affect corporate performance through technological innovation.

Executive equity incentives (EEI) have a positive impact on ROA and are significant at the 1 % significance level. This means that executive equity incentives may not only directly improve corporate performance, but also indirectly improve corporate performance by promoting technological innovation. The conclusions are consistent with the previous article and passed the robustness test.

Considering that there is a lag in the impact of corporate governance and R&D investment on performance, to avoid the endogeneity problem of mutual causation, this paper lags ownership structure Z and technological innovation TI for regression by one period as shown in Table 8 above.

**Table 8:** Endogeneity test.

	(1)	(2)	(3)
	ROE	TI	ROE
L.Z	0.0069**	0.1082***	0.0063**
	(2.3235)	(5.2348)	(2.1377)
L.TI			0.0048**
			(2.4978)
BS	0.0207**	0.1366**	0.0207**
	(2.4715)	(2.3225)	(2.4627)
EEI	0.0005*	0.0055***	0.0004*
	(1.8827)	(3.1948)	(1.7681)
DTAR	0.0099	−0.1218*	0.0111
	(0.9399)	(-1.6479)	(1.0517)
FS	0.0070***	0.6961***	0.0040
	(2.5790)	(36.6079)	(1.3516)
NPGR	0.0023***	−0.0039***	0.0024***
	(13.6842)	(-3.3200)	(13.9066)
_cons	−0.1175**	2.2255***	−0.1369**
	(-2.0073)	(5.4258)	(-2.3194)
N	5373	5373	5373
F	18.0177	605.7665	17.2510
Firm	Yes	Yes	Yes
Year	Yes	Yes	Yes
R^2^	0.0503	0.6404	0.0515

Note: *, **, and *** represent significance at the 10 %, 5 %, and 1 % levels respectively, and the t values are in parentheses.

The article "Corporate governance, technological innovation, and corporate performance: Evidence from China" was retracted in 2025. Reasons: unreliable results or conclusions; concerns about the authorship.

The results are shown in Table 8. As can be seen from Table 8, the regression coefficient of Z in column (1) lags one period is 0.0069, which is significant at the 5 % level. The regression coefficient of BS is 0.0207, which is significant at the 5 % level. The regression coefficient of EEI The coefficient is 0.0005, which is significant at the 10 % level, indicating that after considering endogeneity issues, Z, BS, and EEI can directly promote ROE.

The regression coefficient of Z in column (2) lagged one period is 0.1082, which is significant at the 1 % level. The regression coefficient of BS is 0.1366, which is significant at the 5 % level. The regression coefficient of EEI is 0.0055, which is significant at the 1 % level. is significant, indicating that after considering endogeneity issues, Z, BS, and EEI can directly promote technological innovation.

The regression coefficient of Z in column (3) lagged one period is 0.0063, which is significant at the 5 % level. The regression coefficient of BS is 0.0207, which is significant at the 5 % level. The regression coefficient of EEI is 0.0004, which is significant at the 10 % level. is significant, and the regression coefficient of TI lagged one period is 0.0048, which is significant at the 5 % level, indicating that after considering the endogeneity problem, Z, BS, and EEI can indirectly promote technological innovation through technological innovation, which is consistent with the previous conclusion.

### 4.5 Mediation effect test

Previous research shows that corporate governance has a positive impact on corporate performance. To further examine the mediating role of technological innovation in corporate governance and corporate performance. This article draws on the classic mediation model[63], and sets up the following recursive equations to examine the specific transmission path between the two:

(2) $${\text{ROE}}_{i,t}=a_{0}+a_{1}Z_{i,t}+a_{2}{\text{BS}}_{i,t}+a_{3}{\text{EEI}}_{i,t}+a_{4}{\text{DTAR}}_{i,t}+a_{5}{\text{FS}}_{i,t}+a_{6}{\text{NPGR}}_{i,t}+\sigma_{i,t}+\varepsilon_{i,t}$$

(Equation (2) is set as abovementioned to examine the impact of corporate governance on corporate performance.**)**

(3) $${\text{TI}}_{i,t}=a_{0}+a_{1}Z_{i,t}+a_{2}{\text{BS}}_{i,t}+a_{3}{\text{EEI}}_{i,t}+a_{4}{\text{DTAR}}_{i,t}+a_{5}{\text{FS}}_{i,t}+a_{6}{\text{NPGR}}_{i,t}+\sigma_{i,t}+\varepsilon_{i,t}$$

(Equation (3) is set as abovementioned to examine the impact of corporate governance on technological innovation.)

(4) $${\text{ROE}}_{i,t}=a_{0}+b_{1}{\text{TI}}_{i,t}+a_{1}Z_{i,t}+a_{2}{\text{BS}}_{i,t}+a_{3}{\text{EEI}}_{i,t}+a_{4}{\text{DTAR}}_{i,t}+a_{5}{\text{FS}}_{i,t}+a_{6}{\text{NPGR}}_{i,t}+\sigma_{i,t}+\varepsilon_{i,t}$$

(Equation (4) examines the intermediary effect of technological innovation.)

The article "Corporate governance, technological innovation, and corporate performance: Evidence from China" was retracted in 2025. Reasons: unreliable results or conclusions; concerns about the authorship.

Among them, ROE_i,t_ is corporate performance,Z_i,t_ is equity balance degree, BS_i,t_ is board size, EEI_i,t_ is executive equity incentive, TI_i,t_ is technological innovation, DTAR_i,t_ is the asset-liability ratio、FS_i,t_ is the scale of the corporate, NPGR_i,t_ is the net profit growth rate,σ_i,t_ is the individual and time fixed effects, ε_i,t_ is the random disturbance term.

As shown in Table 9, this study further explores the mediating role of technological innovation (TI) between independent variables (including equity balance degree Z, board size BS, executive equity incentive EEI) and corporate performance (ROE).

**Table 9:** Mediation test.

	(1)
	ROE
TI	0.0223***
	(12.2771)
Z	0.0047*
	(1.7828)
BS	0.0154**
	(2.0513)
EEI	0.0004*
	(1.9204)
DTAR	0.0188**
	(2.0050)
FS	−0.0118***
	(-4.3143)
NPGR	0.0023***
	(14.6076)
_cons	−0.0899*
	(-1.7395)
N	5970
F	26.6003
Firm	Yes
Year	Yes
R^2^	0.0736

Note: *, **, and *** represent significance at the 10 %, 5 %, and 1 % levels respectively, and the t values are in parentheses.

In this study, the coefficient of technological innovation (TI) on ROE is 0.0223, both significant at the 1 % significance level. This shows that technological innovation has a significant positive impact on corporate performance, that is, an increase in the level of technological innovation can significantly increase a company's return on net assets and return on total assets. The direct impact coefficient of equity balances degree(Z) on ROE is significant at the 10 % significance level. This may indicate that part of the impact of equity checks and balances is realized through the intermediary variable of technological innovation. That is, the degree of equity checks and balances may improve corporate performance by promoting technological innovation. Board size (BS) has a positive impact on ROE and is significant at the 5 % significance level. This indicates that board size may directly affect corporate performance, but may also indirectly affect corporate performance through technological innovation. Executive equity incentives (EEI) have a positive impact on ROE and are significant at the 10 % significance level in the model.

The article "Corporate governance, technological innovation, and corporate performance: Evidence from China" was retracted in 2025. Reasons: unreliable results or conclusions; concerns about the authorship.

To sum up, it can be concluded that technological innovation is an important intermediary variable in improving corporate performance. Factors such as ownership structure, board size, and executive equity incentives not only directly affect corporate performance, but may also indirectly affect corporate performance through technological innovation. The mediating effect of Z is 0.0024, the mediating effect of BS is 0.003, and the mediating effect of EEI is 0.0001. These findings have important theoretical and practical significance for understanding how corporate internal governance structures and financial conditions affect corporate performance through technological innovation. Thus, company management behavior profoundly influences enterprise reality across various dimensions, including organizational culture, performance, innovation, financial health, stakeholder relations, and risk management. By fostering a culture of integrity, accountability, and continuous improvement, effective management behavior can drive sustainable success and value creation for the organization and its stakeholders. Stakeholders can actively contribute to or benefit from improved corporate governance and innovation practices. Shareholder activism is very helpful on the greater improvement of work quality and efficiency of top management teams in A-share listed companies in China, the employee participation in innovation processes is also very popular as a good way to utilize the collective wisdom of all employees to make more innovations and improve corporation governance in A-share listed companies in China.

## 5 Discussion

Corporate governance plays an important role in the sustainable development of enterprises. This study uses China's A-share listed companies from 2012 to 2021 as a sample to study the impact of corporate governance on corporate performance and attempts to explore the intrinsic mechanism of the response. The following main conclusions were drawn from the research: (1) Equity balance degree, board size, and executive equity incentives have a positive impact on corporate performance, and the substitution dependent variable method is further used for robustness testing, and the conclusion remains unchanged. (2) Through research on the internal mechanism, it is found that the degree of equity checks and balances, the size of the board of directors, and executive equity incentives are conducive to a company's technological innovation. The higher the technological level of an enterprise, the more conducive it is to improve corporate performance, that is, technological innovation plays an important role in corporate governance (equity balances degree, board size, executive equity incentives) and plays a mediating role in the impact of corporate performance levels.

The article "Corporate governance, technological innovation, and corporate performance: Evidence from China" was retracted in 2025. Reasons: unreliable results or conclusions; concerns about the authorship.

Based on the above research results, during the development process, enterprises should improve the transparency and fairness of corporate governance, protect the legitimate rights and interests of shareholders, directors, executives, employees, etc., strengthen internal and external supervision and restraint mechanisms, and prevent conflicts of interest. and moral hazard, and create a good atmosphere conducive to technological innovation.

Secondly, enterprises should design reasonable incentive mechanisms and strengthen investment and management of technological innovation to improve the efficiency and quality of technological innovation. Companies can use equity incentives to enable managers to create more value for shareholders. It is also possible to implement performance-based pay structures that motivate employees and executives to prioritize and actively participate in technological innovation efforts.

Finally, enterprises should promote the transformation and application of technological innovation, accelerate the industrialization and commercialization of scientific and technological achievements, open up channels for connecting technological innovation and market demand, enhance the market competitiveness and social value of technological innovation, and realize the integration of technological innovation and corporate performance. Performance-Based Compensation: Implementing performance-based compensation structures can incentivize employees and executives to prioritize and actively contribute to technological innovation efforts.

Thus, scientific and technological innovation is crucial for enterprises to gain competitive advantage in the global market. Enterprises can take technological innovation as their core competitiveness to achieve competitive advantage in the global market. Companies should also provide training and support to help employees be creative and innovative, continuously improve the international status of the enterprise.

## 6 Limitations and further research

This study is limited to the research on the impact of internal corporate governance on corporate performance and selects mainly Chinese A-share listed companies to test the roles of technological innovation on corporate performance. The research findings drawn from this paper might have different regulatory or cultural contexts on corporate performance due to different ownership structure or judicial supervision systems on corporate governance, which will be examined in future research.

The article "Corporate governance, technological innovation, and corporate performance: Evidence from China" was retracted in 2025. Reasons: unreliable results or conclusions; concerns about the authorship.

Further studies on the influence mechanism of external corporate governance on corporate performance, and the difference between internal corporate governance and external corporate governance on corporate performance are helpful for a better understanding of the research topic in the future.

## Data availability statement

The data involved in this paper is available on the website at http://www.cninfo.com.cn/new/index, no accession number is necessary.

## Funding & gratitude

The research in this paper was supported by the Scientific Research Program Fund for Higher Schools of the 10.13039/100015790Department of Education of Ningxia Hui Autonomous Region (No. NYG2022105). The authors would like to thank the anonymous reviewers for their many suggestions, which helped to improve the presentation and quality of the paper. The deficiencies in this paper represent the authors' personal views only. Any deficiency in this paper is the responsibility of the authors.

## CRediT authorship contribution statement

**Yinlong Ma:** Writing – original draft, Software, Resources, Project administration, Methodology, Investigation, Formal analysis, Data curation, Conceptualization.

## Declaration of competing interest

The authors declare that they have no known competing financial interests or personal relationships that could have appeared to influence the work reported in this paper.

## References

[1] Bourne M., Franco M., Wilkes J. (2003). Corporate performance management. Measuring Business Excellence.

[2] Kaplan S.N. (1997). Corporate governance and corporate performance: a comparison of Germany, Japan, and the US. Bank Am. J. Appl. Corp. Finance.

[3] Letangule S.L., Letting D., Nicholas K. (2012). Technological innovation and corporate performance. Int. J. Manag. Bus. Stud..

[4] Sui B., Yao L. (2023). The impact of digital transformation on corporate financialization: the mediating effect of green technology innovation. Innovation and Green Development.

[5] Li W.A., Hao C., Cui G.Y., Zheng M.N., Meng Q.K. (2019). Forty years of corporate governance research: a review and agenda. Foreign Economics & Management.

[6] Li S.F., Huang R., Huo W.J., Li Q.J. (2022). Does the leadership of the board of directors affect corporate performance? Based on the empirical research of China's SMEs. Emerg. Mark. Finance Trade.

[7] Feng Y., Chen H., Chen Z.J., Wang Y., Wei W.D. (2021). Has environmental information disclosure eased the economic inhibition of air pollution?. J. Clean. Prod..

The article "Corporate governance, technological innovation, and corporate performance: Evidence from China" was retracted in 2025. Reasons: unreliable results or conclusions; concerns about the authorship.

[8] Pan X.F., Ai B.W., Ming Y. (2019). Research on the spatial spillover effect of interregional technological innovation in China. Oper. Res. Manag. Sci..

[9] Yang L., Qin H., Gan Q., Su J. (2020). Internal control quality, enterprise environmental protection investment and finance performance: an empirical study of China's a-share heavy pollution industry. Int. J. Environ. Res. Publ. Health.

[10] Salehi M., Moradi M., Faysal S. (2023). The relationship between corporate governance and cost of equity: evidence from the ISIS era in Iraq. Int. J. Emerg. Mark..

[11] Sun Y.M. (2020). A study on the impact of shareholding structure on corporate performance based on A-share listed information technology industry. Commercial Accounting.

[12] Wang J.M. (2021). Managing R&D in Chinese listed firms: the interactive effects of ownership concentration and corporate governance [Article]. Thunderbird Int. Bus. Rev..

[13] Yuan Y. (2023). Party organization participation in governance, executive on-the-job spending, and corporate innovation performance. Highlights in business. Econ. Manag..

[14] Liang G.P., Huang Y.Y. (2017). Ownership structure, industry protection, and corporate performance: Empirical data from China A-shares,Finance and Economy.

[15] Chen S.M., Bu M., Wu S.B., Liang X. (2015). How does TMT's attention to the innovation of Chinese firms influence firm innovation activities? A study on the moderating role of corporate governance. J. Bus. Res..

[16] Peng X.H., Zhang R.R. (2022). Corporate governance, environmental sustainability performance, and normative isomorphic force of national culture. Environ. Sci. Pollut. Control Ser..

[17] Moore M.A., Vining A.R. (2023). PPP performance evaluation: the social welfare goal, principal–agent theory, and political economy. Pol. Sci..

[18] Wang L., Pan F. (2023). Incentive mechanism analysis of environmental governance using multitask principal–agent model. Sustainability.

[19] Hu K., Ren Z., Yang J. (2023). Principal-agent problem with multiple principals. Stochastics.

[20] Zheng W., Ding Y.F., Liu D. (2019). 2019 3rd International Seminar on Education, Management and Social Sciences (ISEMSS).

[21] Zhang L., Wang P., Mao D. (2010). The influence of ownership concentration and ownership balance on enterprise performance. Stat. Decis..

[22] Guan B.l., Ge Z.S. (2021). Analysis of the threshold effect of shareholding checks and balances on corporate performance: an empirical analysis based on small and medium-sized listed companies. South China Finance.

[23] Chen Z.L. (2021). Research on the impact of enterprise R&D investment on enterprise growth with ownership structure as the moderating variable. China Journal of Commerce.

The article "Corporate governance, technological innovation, and corporate performance: Evidence from China" was retracted in 2025. Reasons: unreliable results or conclusions; concerns about the authorship.

[24] Yang Q.P. (2022). A study on the correlation between equity structure and corporate performance of GEM-listed companies. China Small & Medium Enterprises.

[25] Tran M., Beddewela E., Ntim C.G. (2021). Governance and sustainability in southeast Asia [article]. Account. Res. J..

[26] Al-Qatanani N., Siam Y.A. (2021). Can ownership structure and board characteristics affect firm performance?. Accounting.

[27] Neralla N.G. (2022). Can corporate governance structure effect on corporate performance: an empirical investigation from Indian companies. Int. J. Discl. Gov..

[28] Ugoani J.N.N. (2020). Effective board management and good corporate performance in Nigerian public liability companies. Indepen. J. Manag. Prod..

[29] Jensen M.C., Meckling W.H. (2019). Corporate Governance.

[30] Yao H.B., Deng Y.L. (2018). Managerial incentives and accounts receivable management policy. Manag. Finance.

[31] Ni Y., Hu Y. (2021). The influence of equity incentive intensity on corporate performance: a case study of A-share listed companies. Jianghan Trib..

[32] Qing H.F., Shao H.M., Su L.C. (2019). The mediating effect of technological innovation on ownership structure and enterprise performance—empirical based on China's GEM-listed manufacturing companies. Sci. Technol. Prog. Policy.

[33] Yang X.J. (2022). Research on the impact of high-tech enterprise ownership structure on innovation investment. Sci-tech Innovation and Productivity.

[34] Guo L.X., Chen C.M. (2010). Research on the relationship between organizational slack and corporate technological innovation performance - an empirical analysis based on panel data of China's manufacturing listed companies. Science of Science and Management of S.& T.

[35] Sahasranamam S., Arya B., Sud M. (2020). Ownership structure and corporate social responsibility in an emerging market. Asia Pacific. J. Manag..

[36] Chindasombatcharoen P., Chatjuthamard P., Jiraporn P., Treepongkaruna S. (2022). Achieving sustainable development goals through board size and innovation. Sustain. Dev..

[37] Zhao J.F., Pongtornkulpanich A., Cheng W.J. (2022). The impact of board size on green innovation in China's heavily polluting enterprises: the mediating role of innovation openness. Sustainability.

[38] Wu J.Y. (2021).

[39] Liu W.H., Wang Z., Wang Z.H., Yu B. (2020). Research on the relationship between board characteristics and technological innovation efficiency of technology-based enterprises. Securit. Mark. Herald.

[40] Zhao G.Y. (2015). Research on the path and effect of equity incentive to improve enterprise technological innovation. Journal of Guangdong University of Finance & Economics.

The article "Corporate governance, technological innovation, and corporate performance: Evidence from China" was retracted in 2025. Reasons: unreliable results or conclusions; concerns about the authorship.

[41] Lu G.Q. (2019). Equity incentive and technological innovation: empirical evidence from listed companies in China. Acad. Bimest..

[42] Ma H., Wan J.Q. (2017). The influence of equity incentive on independent innovation in high-tech enterprises. Journal of Technology Economics.

[43] Jiang S., Long J. (2022). The mechanism path analysis of the influence of executive Equity Incentive on enterprise technological innovation -- Based on the empirical evidence of Chinese Private listed companies. Journal of Jiangxi Normal University (Philosophy and Social Sciences Edition).

[44] Lu T., Dang Y. (2014). Corporate governance and innovation: differences among industry categories. Econ. Res. J..

[45] Wang J., Deng J. (2021). Research on the effect of executive incentive institutional innovation on the cost of equity-evidence from Chinese listed companies. Front. Psychol..

[46] Yuan Q.C., Song X.R. (2022). The impact of equity decentralization on corporate performance - an empirical analysis with corporate innovation as a mediating variable. Productivity Research.

[47] Qin D.Z., Shao H.M., Sun L.C. (2019). The mediating effect of technological innovation on ownership structure and enterprise performance-empirical based on China's GEM-listed manufacturing companies. Sci. Technol. Prog. Policy.

[48] Baum C.F., Lööf H., Stephan A., Viklund-Ros I. (2022). Innovation by start-up firms: the role of the board of directors for knowledge spillovers. Res. Pol..

[49] Amore M.D., Failla V. (2020). Pay dispersion and executive behavior: evidence from innovation. Br. J. Manag..

[50] Xia L., Gao S., Wei J.C., Ding Q.Y. (2022). Government subsidy and corporate green innovation- Does board governance play a role?. Energy Pol..

[51] Brullebaut B., Galia F., Zenou E. Isabelle Allemand, Chen C.C., Zhang X.Y., Xu D.Y., Shao M. (2018). The relationship between corporate governance and sustainable performance. Journal of Jilin Financial Research.

[52] Di H., An J.J., Yao M.F. (2022). Finding the key to the black box of board diversity and firm performance: a mediating effect analysis of technological innovation. Front. Psychol..

[53] Bos‐Brouwers H.E.J. (2010). Corporate sustainability and innovation in SMEs: evidence of themes and activities in practice. Bus. Strat. Environ..

[54] Zuo J.H. (2021). The impact of shareholding structure on corporate performance. Marketing Circles.

[55] Li Z.H., Liao G.k., Albitar K. (2020). Does corporate environmental responsibility engagement affect firm value? The mediating role of corporate innovation. Bus. Strat. Environ..

[56] He H.Y., Wang W.J. (2021). The effect of shareholding concentration on firm performance-agency cost based mediation effect. Sahng Xun.

The article "Corporate governance, technological innovation, and corporate performance: Evidence from China" was retracted in 2025. Reasons: unreliable results or conclusions; concerns about the authorship.

[57] Souther M.E. (2021). Does board independence increase firm value? Evidence from closed-end funds. J. Financ. Quant. Anal..

[58] Zhang M.L. (2017). Management equity incentives, equity checks and balances and corporate performance. Finance and Accounting for International Commerce.

[59] Gibbons M., Johnston R. (1974). The roles of science in technological innovation. Res. Pol..

[60] Lin S.Y., Lai Y.X. (2019). Does corporate governance affect corporate technological innovation? A comparative study based on listed companies in eastern, central and western China. Collect. Essays Finance Econ..

[61] Chen X.D., Tan Y.T., Lin M.X., Zhang G.Y., Ma W.C., Yang S.W., Peng Y.L. (2021). How information technology investment affects green innovation in Chinese heavy polluting enterprises. Front. Energy Res..

[62] Wang X.W., Bai J., Zhang S. (2020). Ownership concentration degree, equity restriction ratio, and enterprise performance—based on the empirical test of listed logistics enterprises from 2009-2018. J. Xi'an Univ. Archit. Technol..

[63] Wen Z.L., Fang J., Xie J.Y., Ouyang J.Y. (2022). Methodological research on domestic intermediary effects. Adv. Psychol. Sci..

[64] Hu A., Yuan X., Fan S., Wang S. (2023). The impact and mechanism of corporate ESG construction on the efficiency of regional green economy: an empirical analysis based on signal transmission theory and stakeholder theory. Sustainability.

[65] Li X.L., Wang Q.J., Huang S., Shi R.B., Han C.L., Gao Y. (2022). The transfer strategy of digital information technology for heterogeneous manufacturers. J. Organ. End User Comput..

[66] Liu J., Li Q.R., Lin C.Y. (2022). Do list companies' technological innovations make institutional investors' “group holdings” more favorable?: based on network-clustering. J. Organ. End User Comput..

[67] Liu L.P., Liu X.X., Guo Z.H., Fan S.S. (2022). An examination of impact of the board of directors capital on enterprises’ low-carbon sustainable development. J. Sens.

